The article "Effect of QSKL on MAPK and RhoA Pathways in a Rat Model of Heart Failure" was published in 2017. Journal: Evid Based Complement Alternat Med.

# Effect of QSKL on MAPK and RhoA Pathways in a Rat Model of Heart Failure

**DOI:** 10.1155/2017/3903898

**Published:** 2017-04-18

**Authors:** Kai Xia, Qiyan Wang, Chun Li, Zifan Zeng, Yong Wang, Wei Wang

**Affiliations:** ^1^Basic Medical College, Beijing University of Chinese Medicine, Beijing 100029, China; ^2^School of Life Sciences, Beijing University of Chinese Medicine, Beijing 100029, China; ^3^Modern Research Center for Traditional Chinese Medicine, Beijing University of Chinese Medicine, Beijing 100029, China

## Abstract

Qishenkeli (QSKL) is one of the Chinese medicine formulae for treating heart failure and has been shown to have an antifibrotic effect. However, the mechanism of its therapeutic effects remains unclear. In this study, we aimed to explore whether QSKL could exert an antifibrotic effect by attenuating ras homolog family member A (RhoA) and mitogen activated protein kinase (MAPK) pathways. Rats were randomly divided into sham group, model group, QSKL group, and positive control group. Heart failure was induced by ligation of the left ventricle anterior descending artery. Cardiac functions were measured by echocardiography and collagen deposition was assessed by Masson staining. Expressions of the key molecules involved in the RhoA and MAPK pathways were also measured. Twenty-one days after surgery, cardiac functions were severely impaired and collagen deposition was remarkable, while QSKL treatment could improve heart functions and alleviate collagen deposition. Further results demonstrated that the effects may be mediated by suppressing expressions of extracellular signal-regulated kinase (ERK) and c-Jun N-terminal kinase (JNK). Moreover, expressions of RhoA, Rho-associated protein kinase 1/2 (ROCK1/2), and phosphorylated myosin light chain (p-MLC) were also downregulated by QSKL compared with the model group. The cardioprotective mechanism of QSKL on heart failure is probably mediated by regulating both the MAPK and RhoA signaling pathways.

## 1. Introduction

Heart failure (HF) is one of the leading causes of death worldwide and myocardial fibrosis is a critical pathological process in the development of HF [1]. Fibrosis is a scarring process that is characterized by the accumulation of fibroblasts and abnormal deposition of extracellular matrix (ECM) proteins, which lead to remodeled cardiac structures and impaired cardiac functions [2]. The effect of fibrosis on impaired cardiac function has been well recognized [3].

The fibroblast is the most important producer of ECM and the main contributor to cardiac fibrosis [4]. Fibroblasts are cells of mesenchymal origin that produce a wide variety of matrix proteins such as collagens I and III [5]. During the cardiac tissue repair process, angiotensin II (Ang II) activated fibroblasts migrate into the damaged area, where they produce and secrete extracellular matrices [6, 7]. Ang II can activate downstream signaling cascades including the ras homolog family member A (RhoA) and mitogen activated protein kinase (MAPK) through angiotensin type 1 receptor (AT-1R) [8]. RhoA stimulates the Rho-associated coiled-coil containing protein kinase (ROCK) which phosphorylates myosin light chain (MLC). Contraction of fibroblasts could be promoted by phosphorylated MLC [9]. G-proteins can also stimulate ras-raf pathway, which in turn activates the MAPK proteins, such as extracellular signal-regulated kinase (ERK) and c-Jun N-terminal kinase (JNK) [10]. When ERK and JNK are phosphorylated, they stimulate the expression of cyclin D and collagen, enhancing proliferation and migration of the fibroblasts [11].

Targeting fibrosis could alleviate the progression of heart failure and efforts have been made to explore the inhibitors of fibrotic pathways. However, only angiotensin-converting enzyme inhibitors (ACEIs), such as fosinopril, and Ang-receptor blockers (ARBs), such as losartan, have been widely used in the clinical treatment of heart failure [12]. Potential therapeutic strategies still need to be explored to effectively inhibit fibrotic progress.

The ancient traditional Chinese medicine (TCM) Qishenkeli (QSKL), which is isolated from 6 widely used Chinese herbs (Radix Astragali Mongolici, Salvia Miltiorrhiza Bunge, Flos Lonicerae, Scrophularia, Radix Aconiti Lateralis Preparata, and Radix Glycyrrhizae), is produced under the China Pharmacopoeia standard of quality control and has been shown to have cardioprotective properties [13, 14]. Studies showed that some traditional Chinese medicines had significant inhibitory effects on myocardial fibrosis [15, 16]. Our previous studies showed that QSKL has been shown to be effective in slowing down the progression of heart failure in HF model of rats [17]. However, the antifibrotic mechanism of QSKL on MAPK and RhoA pathways has not yet been revealed.

In this study, a HF model was induced by ligation of the left anterior descending (LAD) coronary artery in rats. The cardioprotective mechanisms of QSKL were explored by Hematoxylin-Eosin (HE) staining, Masson staining, immunohistochemistry, real-time PCR, and western blotting techniques. The effects of QSKL on the MAPK and RhoA pathways were studied in order to reveal the antifibrotic mechanisms of QSKL and offer an alternative approach for the clinical treatment of myocardial fibrosis.

## 2. Materials and Methods

### 2.1. Animals and Herbs

Studies were performed according to the* Guide for the Care and Use of Laboratory Animals* published by the National Institutes of Health (NIH Publications number 85–23, revised 1996) and the China Physiological Society's* Guiding Principles in the Care and Use of Animals*. Approval was given by the Animal Care Committee of Beijing University of Chinese Medicine. A total of 90 male Sprague-Dawley (SD) rats weighing 220 g ± 10 g in SPF grade were selected (they were purchased from Beijing Vital River Laboratory Animal Technology Co. Ltd.). QSKL consists of 6 Chinese herbs. Radix Astragali Mongolici (460 g), Salvia Miltiorrhiza Bunge (230 g), Flos Lonicerae (160 g), Scrophularia (160 g), Radix Aconiti Lateralis Preparata (140 g), and Radix Glycyrrhizae (90 g) were purchased from Beijing TongRen-Tang Chinese Medicine Co. Ltd. (Beijing, China). The herbs were sent to the traditional Chinese medicine preparation department of the Pharmacy Department of Beijing China-Japan Friendship Hospital for further extraction and preparation. The major extraction steps were as follows. (1) Herbs were boiled in water for one hour and the extract solution was filtered. This process was repeated three times. (2) Water extract was concentrated at high temperature (75°C) and ethanol was added to the concentrated solution. (3) The concentrated solution was precipitated at low temperature (10°C) for 16 hours. (4) The supernatant was concentrated at high temperature (60°C) after alcohol precipitation. (5) The sediment was dried for 5 hours at vacuum degree of −0.1 MPa. (6) The dry material was screened over an 80-mesh sieve for crushing. After preparation, the extracted QSKL was enriched by 5 times. We administered extracted QSKL dissolved in water to rats. To control the quality of the QSKL extract, the fingerprint spectrum was established by the high performance liquid chromatography (HPLC) method, and the typical chromatogram is shown in Figure 1. The daily raw dosage of QSKL administered to the rats was 18.66 g/kg [18, 19]. The concentrated dosage administered to rats was 3.732 g/kg.

### 2.2. HF Model Preparation

HF was induced by the ligation of the left anterior descending artery as previously described [20]. Briefly, 70 rats were anesthetized with 1% pentobarbital sodium (50 mg/kg i.p.) and a left thoracotomy was performed. The pericardium was carefully torn open with tweezers and the left anterior descending artery was ligated with a 5-0 polypropylene suture near the edge of the left atrium. Then, the thorax was closed with 2-0 absorbable silk surgical sutures. After surgery, the rats were given penicillin G (100000 units per rat, i.p.) for three days to prevent infection and the rats were put on an electric blanket until they woke. The live rats were randomly divided into three groups: eleven in the model group, eleven in the QSKL group, and nine in the positive control group. Fosinopril was used as the positive control drug in this study. The other 20 rats in the sham operation group without LAD ligation were also investigated. One day after the operations, the rats in the QSKL group were treated with QSKL for 21 days at a daily dose of 18.66 g/kg and the rats in the positive control group were treated with fosinopril (Bristol-Myers Squibb, China, Series: H19980197) at a daily dose of 1.2 mg/kg. Before administering QSKL to the rats, we prepared the drug solution at the concentration of 0.3732 g/mL. QSKL powder is well soluble in water. Each rat received about 2.2 mL solutions per day. Meanwhile, the rats in the sham operation group and the model group were given the same amount of saline. The overall mortality rate of HF rats during the entire experimental period was about 45%. Of them, 15 rats died during the surgery and 12 rats died the day after the surgery, likely due to acute cardiac failure or lethal arrhythmias. Four rats died during the following days probably due to inflammation or heart failure. Nine rats were randomly chosen in each group for further analysis.

### 2.3. Assessment of Cardiac Function

Echocardiography was performed in the rats anesthetized with 1.5–2% isoflurane (Abraxis BioScience, Richmond Hill, Ontario, Canada) using a Vevo 2100 (Visual Sonics Inc., Toronto, Ontario, Canada) with a 21 MHz probe central frequency scan head. The following parameters were measured by the M-mode images taken from the parasternal short-axis view at the papillary muscle level: left ventricular end-diastolic dimension (LVEDd), left ventricular end-systolic dimension (LVEDs), ejection fraction (EF), and fractional shortening (FS). FS was calculated using the following equation: FS = [(LVEDd − LVEDs)/LVEDd] × 100%.

### 2.4. Measurement of Serum Indicators

Blood was left on the table at room temperature for 30 minutes and then centrifuged for 10 minutes at 3000 rpm. The upper serum was transferred into a new 1.5 mL Eppendorf tube. The level of angiotensin II in the serum was measured by radioimmunoassay. The myocardial enzymes spectrum, including aspartate transaminase (AST), lactate dehydrogenase (LDH), creatine kinase (CK), creatine kinase of muscle-brain type (CKMB), and alpha-hydroxybutyrate dehydrogenase (a-HBDH), was detected by an automatic biochemical analyzer (Toshiba 120, Japan).

### 2.5. Pathological Section Staining

Cardiac tissue was fixed in paraformaldehyde for 24 hours, embedded in paraffin, and cut into 4 *μ*m thick sections. Then, the sections were processed by HE staining. Collagen volume fraction (CVF) was calculated using Image-Pro Plus software after Masson staining: CVF = (area of collagen)/(area of visual field) × 100%. Immunohistochemistry was used to identify the location of collagen I and collagen III. Integrated optical density (IOD) was used to determine the expression levels of collagens I and III. The primary antibodies of collagen I and collagen III are as follows: anti-collagen I rabbit monoclonal antibody (mAb) (Abcam, ab138492) and anti-collagen III mouse monoclonal antibody (Abcam, ab6310). The detecting systems were as follows: Polink-2 Plus® Polymer HRP Detection System, ZSGB-BIO, China, PV-9001, and PV-9002.

### 2.6. Measurement of mRNA Expressions by Real-Time PCR

Cardiac tissue near infarct border zone was lysed by TissueLyser II (Qiagen, Germany). RNA was extracted by TRIzol Reagent (Ambion, Thermo Scientific, USA) and measured by NanoDrop 2000 (Thermo Scientific, USA). The mRNA was transcribed into cDNA in C1000 Thermal Cycler PCR machine (Bio-Rad, USA) with a RevertAid First Strand cDNA Synthesis Kit (Thermo Scientific, USA, lot number: K1622). The reaction volume was 20 *μ*L including 2 *μ*L of cDNA, 1 *μ*L of forward and reverse primer pairs, 10 *μ*L of FastStart Universal SYBR Green Master (Roche, Germany, lot number: 04913914001), and 7 *μ*L of RNase-free water. The real-time PCR procedures were as follows: 15 s at 95°C for denaturation, followed by 1 min at 60°C for annealing and extension. Each reaction was performed for 40 cycles and Ct values were obtained. Sequences of primers are listed in Table 1. Ct values of targeted mRNA including extracellular signal-regulated kinase (ERK), c-Jun N-terminal kinase (JNK), RhoA, Rho-associated protein kinase 1 (ROCK1), ROCK2, and myosin light chain (MLC) were normalized according to the Ct values of GAPDH. Relative expression levels of these genes were calculated by the 2^−ΔΔCT^ method.

### 2.7. Measurement of Protein Expressions by Western Blot

Proteins were extracted using RIPA buffer (50 mM Tris-HCl, pH 7.4, 150 mM NaCl, 1% NP-40, and 0.1% SDS), cOmplete Tablet EASYpack protease inhibitor (Roche, Germany, lot number: 04693116001), and PhosSTOP EASYpack phosphatase inhibitor (Roche, Germany, lot number: 04906845001). The concentration of each sample was measured by a Spectra Max i3x microplate reader (Molecular Devices, USA) with a protein assay kit (Beijing PuLilai Gene Technology Co., Ltd., Beijing, China, lot number: P1511) and the concentration was adjusted to equal concentration with 5x SDS-PAGE sample buffer. All of the samples were boiled for 5 min. After that, samples were loaded on a 10% SDS-PAGE gel (40 *μ*g protein/10 *μ*L per well) and electrophoresis was performed using PowerPac Universal Power Supply (Bio-Rad, USA) at 100 V for 2 h. Proteins on the gel were transferred onto a nitrocellulose membrane (Pall Corporation, USA) and electrophoresed at 300 mA for 90 minutes. The membrane was first probed with a primary antibody and a secondary antibody (HRP-goat anti-rabbit IgG (H + L), GXYbio, China, S8002); then, it was treated with Amersham ECL prime western blotting detection reagent (GE Healthcare, USA) for 1 min at room temperature. The membrane was exposed in the Molecular Imager ChemiDoc XRS+ System (Bio-Rad, USA), and then the bands on the membrane were visualized and analyzed by Image Lab software. Blot densities of ERK, JNK, phosphorylated ERK (p-ERK), phosphorylated JNK (p-JNK), RhoA, ROCK1, ROCK2, MLC, phosphorylated MLC (p-MLC), and GAPDH were obtained by the same procedure. The primary antibodies were as follows: Phospho-p44/42 MAPK (ERK 1/2) XP® Rabbit mAb, CST, 4370S; Phospho-SAPK/JNK Rabbit mAb, CST, 4668S; ROCK1 Rabbit mAb, CST, 4035S; ROCK2 Rabbit mAb, CST, 9029S; RhoA Rabbit mAb, CST, 2117S; p44/42 MAPK (ERK 1/2) Rabbit mAb, CST, 4695S; SAPK/JNK Antibody, CST, 9252S; Anti-Myosin Light Chain 2 Antibody, Abcam, ab92721; Anti-Myosin Light Chain (phospho-S20) antibody, Abcam, ab2480; GAPDH XPx Rabbit mAb, CST, 5174S. Results of ERK, JNK, RhoA, ROCK1, ROCK2, and MLC were normalized by GAPDH density while the results of p-ERK, p-JNK, and p-MLC were normalized by ERK, JNK, and MLC, respectively.

### 2.8. Statistical Analysis

All of the data are presented as mean ± standard deviation (SD). Statistical analysis was performed by SPSS 20.0 software. Results were carried out using one-way analysis of variance (ANOVA) and Dunnett and Dunnett T3 test. The value of* P* < 0.05 was considered to be statistically significant.

## 3. Results

### 3.1. Effect of QSKL on Cardiac Functions

Compared with the sham group, the LVEDd and LVEDs of the model group were increased by 21.71% (*P* < 0.01) and 113.93% (*P* < 0.01), respectively, suggesting that ventricular hypertrophy had developed in the model rats. Meanwhile, EF and FS were decreased by 63.00% (*P* < 0.01) and 76.98% (*P* < 0.01), respectively, which indicated that cardiac functions were severely damaged and the heart failure had developed in the model rats (Figure 2(b)). After treatment with QSKL, EF and FS were increased by 67.80% (*P* < 0.01) and 133.39% (*P* < 0.01), respectively, compared with the model group (Figures 2(c) and 2(d)). The positive drug fosinopril showed no significant effect on EF or FS. The results showed that QSKL could improve heart functions and inhibit cardiac hypertrophy.

### 3.2. Effect of QSKL on Serum Indicators of Heart Functions

The increase of some serum indicators, such as Ang II, AST, LDH, CKMB, CK, and a-HBDH, could reflect the alteration of cardiac functions. Compared with the sham group, the levels of Ang II, AST, LDH, CKMB, CK, and a-HBDH of the model group were increased by 119.13% (*P* < 0.01), 46.80% (*P* < 0.01), 37.84% (*P* < 0.01), 62.15% (*P* < 0.01), 37.67% (*P* = 0.016), and 36.72% (*P* = 0.018), respectively. After treatment with QSKL, the serum levels of Ang II, AST, LDH, CKMB, CK, and a-HBDH were decreased by 39.34% (*P* < 0.01), 26.53% (*P* < 0.01), 20.46% (*P* = 0.021), 34.15% (*P* = 0.013), 21.80% (*P* = 0.145), and 25.18% (*P* = 0.089), respectively, as compared with the model group. The positive drug fosinopril also downregulated the serum levels of these enzymes in a similar way (Figure 3). These results further suggested that QSKL had a cardioprotective effect under ischemic stimulus.

### 3.3. Effect of QSKL on Cardiac Structures

HE staining showed that the myocardial cells of the sham group were arranged in an orderly way, and the nuclei structures were intact. In contrast, the cells of the model group lost their normal structures and were disorderly arranged. Cardiac fibers were dissolved and necrotized, with the infiltration of many inflammatory cells (Figure 4(b)). In the QSKL treatment group, the cellular structure was arranged more regularly, with less infiltration of inflammatory cells, compared with the model group (Figure 4(c)).

### 3.4. Effect of QSKL on Myocardial Fibrosis and Collagen Deposition

Masson staining was applied to assess the myocardial fibrosis. As shown in Figure 5, there was little interstitial collagen deposition in the sham group. However, extensive collagen deposition, as indicated by blue stains, was observed in the model group. In the QSKL and fosinopril groups, collagen deposition was inhibited as compared with the model group. The collagen volume fraction (CVF) was further quantified. Compared with the sham group, the CVF of the model group was increased by 257.03% (*P* < 0.01). After treatment with QSKL, the CVF were decreased by 36.55% (*P* < 0.01), suggesting that QSKL could effectively attenuate collagen synthesis (Figure 5). Fosinopril also suppressed collagen synthesis, and there was no significant difference between the two groups (Figure 5).

Collagens I and III were assessed by immunohistochemistry. Integrated optical densities (IOD) of collagens I and III in the model group were increased by 277.30% (*P* < 0.01) and 191.06% (*P* < 0.01), respectively, as compared with the sham group. After treatment with QSKL, the IOD of collagens I and III was decreased by 47.33% (*P* < 0.01) and 38.07% (*P* < 0.01), respectively, indicating that QSKL could attenuate the biosynthesis of collagens I and III (Figures 6 and 7). The positive control drug fosinopril also suppressed the synthesis of collagens I and III.

### 3.5. Effect of QSKL on the MAPK Signaling Pathway

Activation of the MAPK signaling pathway promotes development of fibrosis [21]. Compared with the sham group, the mRNA expressions of ERK and JNK in the model group were increased by 464.23% (*P* < 0.01) and 299.93% (*P* < 0.05), respectively. After treatment with QSKL, the mRNA expressions of ERK and JNK were decreased by 62.44% (*P* < 0.01) and 77.04% (*P* < 0.01), respectively. The positive drug fosinopril also suppressed the expressions of ERK and JNK (Table 2). The protein expressions of ERK, JNK, and their phosphorylated forms were also detected by western blotting. Compared with the sham group, the protein levels of ERK, p-ERK/ERK, JNK, and p-JNK/JNK in the model group were increased by 116.69% (*P* < 0.01), 166.71% (*P* < 0.01), 34.50% (*P* = 0.065), and 71.30% (*P* = 0.025), respectively. In the QSKL treatment group, the protein levels of ERK, p-ERK/ERK, JNK, and p-JNK/JNK were downregulated by 58.07% (*P* < 0.01), 37.27% (*P* < 0.05), 29.00% (*P* < 0.05), and 46.11% (*P* < 0.05), respectively, compared with those in the model group (Figure 8). Fosinopril had similar effects on these molecules as QSKL did. Taken together, these results indicated that QSKL had an inhibitory effect on the expressions of ERK and JNK in the MAPK signaling pathway.

### 3.6. Effect of QSKL on the RhoA/ROCK Signaling Pathway

Expressions of key molecules in RhoA/ROCK signaling pathway were evaluated. The mRNA expressions of RhoA, ROCK1, ROCK2, and MLC in the model group were increased by 777.46% (*P* < 0.01), 349.73% (*P* < 0.01), 194.71% (*P* < 0.05), and 69.82% (*P* < 0.01), respectively, compared with the sham group. In the QSKL group, the mRNA expressions of RhoA, ROCK1, ROCK2, and MLC were reduced by 60.39% (*P* < 0.05), 68.65% (*P* < 0.05), 63.25% (*P* < 0.05), and 12.84% (*P* = 0.620), respectively, compared with the model group (Table 3). Fosinopril also downregulated the expression of these molecules. Protein levels of RhoA, ROCK1, ROCK2, MLC, and p-MLC/MLC in the model group were increased by 156.64% (*P* < 0.01), 167.26% (*P* < 0.01), 82.03% (*P* < 0.01), 6.80% (*P* = 0.813), and 83.90% (*P* < 0.01), respectively, as compared with those in the sham group, which indicated that the RhoA/ROCK signaling cascade was activated in the model group. Protein levels of RhoA, ROCK1, ROCK2, MLC, and p-MLC/MLC were downregulated by 47.04% (*P* < 0.01), 56.07% (*P* < 0.01), 41.39% (*P* < 0.01), 2.13% (*P* = 0.990), and 44.30% (*P* < 0.01), respectively, after treatment with QSKL (Figure 9). These results suggested that QSKL could attenuate the activation of RhoA/ROCK signaling cascade during the process of fibrosis.

## 4. Discussion

In this study, we explored the antifibrotic mechanisms of QSKL in the treatment of heart failure. Our main findings include the following. (1) QSKL restored the heart functions that were impaired by ischemic stimuli. The serum indictors of heart damage were restored towards normal levels. (2) Cardiac cellular damage was attenuated by QSKL and extracellular collagen deposition was suppressed by QSKL. (3) The expressions of ERK and JNK were inhibited by QSKL. (4) The RhoA/ROCK signaling pathway was suppressed by QSKL. Our study suggested that the antifibrotic effect of QSKL was probably mediated by suppressing the MAPK and RhoA/ROCK signaling pathways.

QSKL is composed of six herbs. The dosage prescribed to patients in clinic is 1.33 g/kg. The effective components of QSKL can be extracted and concentrated. If QSKL extract is prescribed to patients, the dosage is 0.27 g/kg. The equivalent raw dosage in rats taking into consideration the animal body surface area should be 9.33 g/kg (1.33 times 7) [18, 19]. As the rat's drug tolerance is higher than that of human, we therefore selected 4.67 g/kg, 9.33 g/kg, and 18.66 g/kg as raw dosages in our preexperiments to test the effects of QSKL. The results showed that 18.66 g/kg was the most effective. Therefore, this dosage was chosen in this study. Accordingly, the dosage of extracted QSKL administered to rats was 3.73 g/kg. QSKL has been shown to be effective in slowing down the progression of heart failure by in vivo studies [17, 22, 23]. Exploring the mechanism of QSKL would provide insight into the therapeutic approaches in the management of heart failure. In this study, we induced a rat model of heart failure. The echocardiography results showed that the cardiac function in the QSKL group was remarkably improved compared with the model group, and the HE staining showed that the myocardial damage was alleviated by the QSKL treatment. Deposition of collagens I and III was significantly reduced by QSKL. These results confirmed that QSKL has cardioprotective and antifibrotic effects. We further explored the cardioprotective mechanisms of QSKL in our following studies.

Fibrosis is a prominent pathological characteristic in the progression of heart failure and Ang II has been shown to play an important role in promoting cardiac remodeling [24]. Ang II combines with angiotensin type 1 receptor (AT-1R) and activates the downstream signaling network including the RhoA and MAPK pathways [25]. AT-1R is a G-protein coupled receptor that can interact with small G-proteins, such as RhoA [26]. After receiving the signals from AT-1R, RhoA can combine with GTP and activate the target proteins, such as ROCK1 and ROCK2. The activation of ROCK1/2 will phosphorylate MLC and stimulate the assembling and moving of myosin II, therefore promoting the formation of the contractile ring that enhances cytoplasmic division during the proliferation of the fibroblasts [27, 28]. Meanwhile, the phosphorylation of MLC promotes the turnover of focal adhesion plaques and cell tail contraction, which can elevate the mobility of fibroblasts [29]. Expressions of RhoA, ROCK1, ROCK2, and p-MLC were investigated in this study. In the model group, the mRNA and protein expressions of these molecules were increased, suggesting that the RhoA/ROCK pathway was activated during the cardiac remodeling process. In QSKL treatment group, the expressions of these key molecules were suppressed compared with the model group, indicating that QSKL exerts an antifibrotic effect by blocking the RhoA/ROCK pathway. This inhibitory effect on RhoA/ROCK could be exerted by the effective components of QSKL. Salvianolic acid B, one of the major effective constituents identified in Salvia Miltiorrhiza Bunge, has been shown to inhibit the RhoA signaling pathway in cirrhotic rats [30]. Other components of QSKL, such as astragaloside IV, luteolin, and tanshinone IIA, have also been shown to have inhibitory effects on the RhoA/ROCK pathway under various pathological conditions [31–34].

The MAPK signaling pathway, another pathway activated by RhoA, also plays important roles in the proliferation of fibroblasts [35]. RhoA can activate raf, and the raf will stimulate MEK which phosphorylates the ERK and JNK proteins [36]. Phosphorylated ERK and JNK activate transcription factors such as c-Fos and c-Jun, which then translocate into the nucleus and stimulate gene expression [37, 38]. The expressions of collagen and cyclin D1 are stimulated by the activation of ERK and JNK, promoting the proliferation of fibroblasts and the progression of fibrosis [39, 40]. ERK can also promote fibroblast migration by stimulating the contraction of the cell tail [41]. Our results showed that the expressions of phosphorylated ERK and JNK in the model group were increased and the treatment with QSKL attenuated the expression of these two proteins, suggesting that the MAPK signaling pathway is also a target of QSKL in the treatment of heart failure. A previous study showed that liquiritin, the major constituent of Radix Glycyrrhizae, could suppress diabetes-related myocardial fibrosis by suppressing the MAPK pathway [42]. Salvianolic acid B has also been shown to have inhibitory effects on the MAPK pathway in several studies [43–45]. Fosinopril, an angiotensin-converting enzyme inhibitor, was applied as the positive control drug in this study and it showed similar effects on the RhoA/ROCK pathway. However, the cardioprotective effect of QSKL was more remarkable than that of fosinopril. In addition, the protein levels of p-ERK and JNK in the QSKL group were downregulated more significantly compared with the fosinopril group. Taken together, our study suggests that QSKL exerts an antifibrotic effect in a multitarget mode and QSKL is an ideal alternative in the treatment of heart failure.

## 5. Conclusions

QSKL exerts cardioprotective effects by inhibiting the progression of fibrosis in a heart failure model. The antifibrotic mechanism is probably mediated by suppressing the RhoA/ROCK and MAPK signaling pathways (Figure 10). Targeting key molecules in the Ang II-AT1R-RhoA pathway could offer an alternative therapeutic approach in the management of myocardial fibrosis.

## Figures and Tables

**Figure 1:** HPLC chromatogram of QSKL at 254 nm. 1: chlorogenic acid; 2: cryptochlorogenic acid; 3: neochlorogenic acid; 4: secologanic acid; 5: sweroside; 6: Secoxyloganin; 7: liquiritin; 8: isochlorogenic acid A; 9: isochlorogenic acid C; 10: ononin; 11: salvianolic acid B; 12: calycosin; 13: harpagoside; 14: formononetin; 15: glycyrrhizic acid.

**Figure 2:** QSKL improved cardiac functions (*n* = 9). Parameters of cardiac functions were detected by echocardiography. (a) shows that LVEDd, LVEDs, EF, and FS were normal in the sham group. (b) shows that LVEDs were upregulated, while EF and FS were downregulated in the model group compared with the sham group. (c) shows that EF and FS were upregulated in the QSKL group compared with those in the model group. (d) shows that there was a modest improvement of EF and FS in the fosinopril group (^*∗*^*P* < 0.05, ^*∗∗*^*P* < 0.01, other groups versus model group).

**Figure 3:** Effects of QSKL on the serum indicators (*n* = 9). Plasma levels of Ang II, AST, LDH, CKMB, CK, and a-HBDH in the four groups of rats were detected by a biochemical analyzer. QSKL could decrease Ang II, AST, LDH, and CKMB levels compared with the model group. Levels of CK and a-HBDH showed no statistical difference between the QSKL group and the model group. Fosinopril had a similar effect to QSKL (^*∗*^*P* < 0.05, ^*∗∗*^*P* < 0.01, other groups versus model group).

**Figure 4:** Effects of QSKL on the cardiac structures detected by HE staining. When observed under the magnification of 200x, (a) shows that the myocardial cells of the sham operation group were arranged in an orderly way. In contrast, (b) shows that the cells of model group lost their normal structures. Cardiac fibers were dissolved and necrotized, with infiltration of many inflammatory cells. (c) and (d) show that cells were arranged in a much orderly way and there were fewer inflammatory infiltrations in the QSKL and positive control group.

**Figure 5:** Effects of QSKL on collagen deposition (*n* = 9). Collagen was stained blue by Masson staining. When observed under the magnification of 200x, (a) shows that there was little deposition of collagen among cardiac cells. (b) showed that there was extensive deposition of collagens in the model group. (c) and (d) showed that collagens were reduced in QSKL and fosinopril groups as compared with those in the model group. Compared with sham group, the CVF values in the model group were upregulated, and QSKL could decrease the CVF value compared with model group (^*∗*^*P* < 0.05, ^*∗∗*^*P* < 0.01, other groups versus model group).

**Figure 6:** Deposition of collagen I was assessed by immunohistochemistry (*n* = 9). (a) shows that there was little deposition of collagen I in the sham group. (b) shows that there was extensive deposition of collagen I in the model group. (c) and (d) show that the amount of collagen I in the QSKL group and fosinopril group was much less as compared with the model group. Compared with the sham group, the IOD value of collagen I in the model group was upregulated. QSKL could decrease the IOD value of collagen I compared with the model group. The level showed no statistical difference between the fosinopril group and the QSKL group (^*∗*^*P* < 0.05, ^*∗∗*^*P* < 0.01, other groups versus model group).

**Figure 7:** Deposition of collagen III was assessed by immunohistochemistry (*n* = 9). (a) shows that there was little deposition of collagen III in the sham group. (b) shows that there was extensive deposition of collagen III in the model group. (c) and (d) showed that QSKL and fosinopril suppressed expression of collagen III compared with the model group. Compared with the sham group, the IOD value of collagen III in the model group was upregulated. QSKL could decrease the IOD value of collagen III compared with the model group. The level showed no statistical difference between the fosinopril group and the QSKL group (^*∗*^*P* < 0.05, ^*∗∗*^*P* < 0.01, other groups versus model group).

**Figure 8:** Effects of QSKL on the MAPK pathway (*n* = 9). Western blot shows that the expressions of ERK, p-ERK, and p-JNK in the model group were upregulated compared with the sham group. QSKL could decrease levels of ERK, p-ERK/ERK, JNK, and p-JNK/JNK compared with the model group. Levels of p-ERK and JNK showed no statistical difference between the fosinopril group and the model group (^*∗*^*P* < 0.05, ^*∗∗*^*P* < 0.01, other groups versus model group).

**Figure 9:** Effects of QSKL on the RhoA/ROCK pathway (*n* = 9). Western blot shows that the expressions of RhoA, ROCK1, ROCK2, and p-MLC/MLC in the model group were upregulated compared with the sham group. QSKL could decrease the levels of RhoA, ROCK1, ROCK2, and p-MLC/MLC compared with the model group. Level of MLC showed no statistical difference between the fosinopril group and the model group (^*∗*^*P* < 0.05, ^*∗∗*^*P* < 0.01, other groups versus model group).

**Figure 10:** Antifibrosis mechanisms of QSKL on the RhoA/ROCK and MAPK pathways. The RhoA/ROCK and MAPK pathways contribute to fibrosis by promoting the migration and proliferation of fibroblasts. During the fibrotic process, Ang II combines with AT-1R, which can interact with G-proteins such as RhoA. After receiving a signal from AT-1R, RhoA will activate the target proteins, such as ROCK1 and ROCK2, which in turn phosphorylate MLC and enhance the cytoplasmic division during fibroblast proliferation. Meanwhile, MLC promotes cell migration by accelerating the turnover of focal adhesion plaques. RhoA can also activate the raf protein on the upper stream of the MAPK signaling pathway. Activated raf stimulates MEK which then phosphorylates the ERK and JNK proteins. Phosphorylated ERK and JNK activate certain transcription factors that translocate into the nucleus and stimulate fibroblast proliferation. QSKL inhibits the proliferation and migration of the fibroblasts by acting on the key molecules in the RhoA/ROCK and MAPK signaling pathways, thereby exerting antifibrosis effects.

**Table 1:** Nucleotide sequences of primers used in real-time PCR.

Gene	Primers	Nucleotide sequences 5′-3′	Length (bp)	Temp. (°C)
ERK	Forward	AAAAGGGGGAGGGGACGTAA	87	60.5
	Reverse	CCACTCACCTGTTTCCTGTCT		59.6
JNK	Forward	GCCTGGACTGTGACGTCTATTT	195	60.2
	Reverse	AGCATTCCCTACAAAGTGCC		58.7
RhoA	Forward	TGTTTTTCCATCGACAGCCCT	171	60.2
	Reverse	TACCGGCTCCTGCTTCATTT		59.4
ROCK1	Forward	ACCTTCTGGCTTTGTCCGT	159	59.2
	Reverse	CCTGGTGATCAGGTAGCAT		57.4
ROCK2	Forward	TCCCTTCCCTGTGGTGACTT	88	60.4
	Reverse	GGGAAAGGAGCTGGTTCAAGA		59.9
MLC	Forward	TCGACGCCATGATGAAGGAA	200	59.5
	Reverse	CTGGGAAAATCGGTCGCACT		60.7
GAPDH	Forward	ATTCCATCCCAGACCCCATAAC	81	59.5
	Reverse	GCAGCGAACTTTATTGATGGTAT		57.6

**Table 2:** mRNA expression of ERK and JNK in four different groups of rats.

Group	Sham	Model	QSKL	Fosinopril
ERK	1.00 ± 0.54^*∗∗*^	5.64 ± 1.53	2.12 ± 0.76^*∗∗*^	1.45 ± 0.38^*∗∗*^
JNK	1.00 ± 0.12^*∗*^	4.00 ± 0.64	0.92 ± 0.18^*∗∗*^	0.97 ± 0.12^*∗*^

Data were presented as mean ± standard deviation (*n* = 9). Compared with the model group, ^*∗*^*P* < 0.05 and ^*∗∗*^*P* < 0.01.

**Table 3:** mRNA expression of key molecules in the RhoA/ROCK pathway in four different groups of rats.

Group	Sham	Model	QSKL	Fosinopril
RhoA	1.00 ± 0.19^*∗∗*^	8.77 ± 3.93	3.48 ± 0.89^*∗*^	3.05 ± 0.72^*∗*^
ROCK1	1.00 ± 0.09^*∗∗*^	4.50 ± 1.95	1.41 ± 0.31^*∗∗*^	1.38 ± 0.33^*∗∗*^
ROCK2	1.00 ± 0.11^*∗*^	2.95 ± 1.34	1.08 ± 0.11^*∗*^	1.06 ± 0.10^*∗*^
MLC	1.00 ± 0.47^*∗∗*^	1.70 ± 0.58	1.48 ± 0.35	1.32 ± 0.23

Data were presented as mean ± standard deviation (*n* = 9). Compared with the model group, ^*∗*^*P* < 0.05 and ^*∗∗*^*P* < 0.01.
